The article "Effects of Acupuncture on Cortical Activation in Patients with Disorders of Consciousness: A Functional Near-Infrared Spectroscopy Study" was published in 2022. Journal: Evid Based Complement Alternat Med.

# Effects of Acupuncture on Cortical Activation in Patients with Disorders of Consciousness: A Functional Near-Infrared Spectroscopy Study

**DOI:** 10.1155/2022/5711961

**Published:** 2022-07-14

**Authors:** Xin Wen, Zicai Liu, Yuchun Shao, Yang Peng, Huiyu Liu, Minghong Wang, Junbin Chen

**Affiliations:** ^1^Department of Rehabilitation Medicine, Yue Bei People's Hospital, Shaoguan, Guangdong, China; ^2^Gannan Medical University, Ganzhou, Jiangxi, China; ^3^Department of Neurology Medicine, Yue Bei People's Hospital, Shaoguan, Guangdong, China

## Abstract

**Background:**

Disorder of consciousness (DoC) is a clinical condition caused by severe brain damage. Some studies have reported that acupuncture, a traditional Chinese treatment, could facilitate the recovery of the patient's consciousness. The therapeutic effects of acupuncture may be due to its modulation of facilitating cortex (PFC) activity, but it has not been greatly demonstrated.

**Objectives:**

We intended to observe the effects of acupuncture on prefrontal cortical activity, explore the potential correlation between cortical activation and the severity of DoC, and analyze the functional brain network connectivity to provide a theoretical basis for its application in clinical practice.

**Methods:**

Participants diagnosed with DoC were included in the study. Before the intervention, we assessed the patient's state of consciousness using relevant scales, such as the Glasgow coma scale (GCS) and the coma recovery scale-revised (CRS-R). All patients received acupuncture manipulation with the functional near-infrared spectroscopy (fNIRS) system monitored.

**Result:**

A total of 16 subjects participated in our study. We observed that the concentration of oxygenated hemoglobin (HbO) in the PFC was increased during the acupuncture manipulation and declined during the resting state. Then, the connection strength of the left cerebral cortex was generally higher than that of the right. Finally, we observed only a weak difference in hemodynamic responses of PFC between the vegetative state (VS) and minimally conscious state (MCS) groups. However, the difference was not statistically significant.

**Conclusion:**

Our results indicated that acupuncture can increase the concentration of HbO in the PFC and strengthen the connection strength of the left cerebral cortex. However, our present study did not find a significant correlation between the cortical hemodynamic response and the severity of DoC.

## 1. Introduction

A disorder of consciousness (DoC) is a state in which there is a disturbance in the way people perceive themselves and their environment or in the mental activities by which they perceive their environment. Many diseases can lead to impaired consciousness, such as cerebral infarction, cerebral hemorrhage, and traumatic brain injury (TBI) [1]. DoC contains coma, vegetative state (VS), and minimally conscious state (MCS) [2, 3]. Coma is the most serious DoC where the patient cannot be awakened and is without a normal sleep-wake cycle [4]. VS, also named unresponsive wakefulness syndrome (UWS), is when the patient can open their eyes but is unresponsive (i.e., only shows reflexive movements and does not respond to commands) [5]. Patients with MCS can perceive their environment consciously and respond repetitively to environmental stimuli [6–8]. The main mechanisms for the occurrence of consciousness disorders are cerebral ischemia, hypoxia, inadequate glucose supply, and abnormal enzyme metabolism, which can cause metabolic disorders in brain cells, thus leading to impairment of reticular structure function and brain hypofunction [9]. Patients with consciousness disorders are bedridden for long periods, unable to care for themselves, and expensive to treat. This is a huge burden and has an impact on the family and society, so it is very necessary to facilitate the recovery of the patient's conscious state.

The article "Effects of Acupuncture on Cortical Activation in Patients with Disorders of Consciousness: A Functional Near-Infrared Spectroscopy Study" was published in 2022. Journal: Evid Based Complement Alternat Med.

Some studies have shown that acupuncture could improve blood circulation to the brain, promote the recovery and regeneration of brain nerve cells, stimulate nerve cells in a “dormant” state, and relieve cortical inhibition, thus facilitating the recovery of the patient's state of consciousness [10]. Renzhong point (GV26) is one of the common acupuncture points to improve consciousness disorders. It is located at the junction of the upper 1/3 and middle 1/3 of the Renzhong sulcus [11] and has the effect of tranquilizing and calming the mind, awakening the brain, and opening the orifices [12]. The acupuncture technology mainly includes needle liftings and needle twists. A study by Li et al. [13] found that acupuncture of the Renzhong acupoint significantly increased cerebral blood flow and dilated microvascular diameter, which in turn improved impaired consciousness.

Functional near-infrared spectroscopy (fNIRS) is a substitutable tool for fMRI with features such as noninvasiveness and portability, and it can instantly respond to the activity of the cerebral cortex by detecting the concentration changes of oxygenated hemoglobin (HbO) and deoxygenated hemoglobin (HbR) in the target cortical region [14, 15]. Laureys and Schiff [16] proposed a model of consciousness as a collective behavior of extensive prefrontal network connections regulated by specific brain circuit mechanisms. Compared with other technologies (fMRI and EEG), fNIRS is safe, portable, and relatively inexpensive, making it convenient to implement [17, 18].

The article "Effects of Acupuncture on Cortical Activation in Patients with Disorders of Consciousness: A Functional Near-Infrared Spectroscopy Study" was published in 2022. Journal: Evid Based Complement Alternat Med.

Therefore, based on the above background, the purpose of this experiment is to use fNIRS to detect the concentration changes of HbO in the prefrontal cortex (PFC), to compare concentrations of HbO during acupuncture and resting state in patients with DoC, to explore the potential correlation between the prefrontal cortical hemodynamic response and the severity of patients' impaired consciousness, and to analyze the functional brain network connectivity to provide a theoretical basis for its application in clinical practice.

## 2. Materials and Methods

### 2.1. Participants

All patients were recruited from the Department of Rehabilitation Medicine and Neurology Medicine, Yuebei People's Hospital, between June 2021 and September 2021. Subjects included in the trial met the following inclusion criteria: aged >18 years; all patients met the diagnostic criteria for DoC, referring to the European Academy of Neurology guidelines for the diagnosis of coma and other disorders of consciousness in 2020 [4]; vital signs were stable; and family members voluntarily signed an informed consent form. The exclusion criteria were as follows: (1) intracranial retention of metal objects, cranial debridement, or presence of cranial defects and any clinically significant or unstable medical disorders. All subjects signed an informed consent form before enrollment in the study. The experiment was supported by the Human Research Ethics Committee of Yuebei People's Hospital (number: KY-2021-095), and our clinical trial was conducted and reported in accordance with the Consolidated Standards for Reporting Trials (CONSORT) guidelines [19]. The protocol was registered with the China Clinical Trials Registry under the registration number: ChiCTR2100051970.

### 2.2. Methods

The traditional Chinese acupuncture techniques were used in this experiment, and all procedures were completed by a professional acupuncturist. The experiment comprised 3 tasks: needle insertion, needle twirls, and needle removal. Methods and procedures were followed according to the 2019 study by Fernandez Rojas et al. [18].

The first task is a 5s insertion needle after a 5s preparation. The second task is a 30s needle twirl after resting for 30S and then repeated twice again. The third task is a 5S needle removal. The entire manipulation process is shown in Figure 1. The acupoint utilized in our trial was the Renzhong point. We chose the Renzhong point because it is the most frequently used point to improve consciousness disorders and promote wakefulness. All patients were detected with the fNIRS system in the supine position.

The article "Effects of Acupuncture on Cortical Activation in Patients with Disorders of Consciousness: A Functional Near-Infrared Spectroscopy Study" was published in 2022. Journal: Evid Based Complement Alternat Med.

### 2.3. Assessment

All subjects were assessed by the fNIRS system and scales related to the impairment of consciousness, including the Glasgow coma scale (GCS) and the coma recovery scale-revised (CRS-R).

#### 2.3.1. Glasgow Coma Scale (GCS)

The GCS is extensively applied to objectively describe the severity of DoC [20]. The scale consists of three aspects: eye-opening response (E), verbal response (V), and motor response (E), with a maximum score of 15 and a minimum score of 3 [21]. Standards of evaluation: 15 points indicate clear consciousness; 12–14 points indicate mildly impaired consciousness; 9–11 points indicate moderately impaired consciousness; and less than 9 points indicate coma. The lower the score, the more severe the DoC.

#### 2.3.2. Coma Recovery Scale-Revised (CRS-R)

The CRS-R is an established tool and is widely acknowledged as the international gold standard for the behavioral assessment of diagnoses of DoC [22–24]. The CRS-R is composed of six subscales for auditory, verbal, visual, communication, motor, and arousal levels [25]. The scale score ranges from 0 to 23 [26], with higher scores resulting in lower levels of impaired consciousness. The scale was developed specifically to distinguish between MCS and VS [23, 27], and the specific evaluation criteria [27] are given in Table1.

The GCS and CRS-R assessments were implemented by two professional physicians in rehabilitation. Any differences in the evaluation process were resolved through discussion. Subjects were grouped into VS and MCS groups according to their CRS-R scores. Based on the GCS score, subjects were divided into moderate DoC and severe DoC groups. The patient subgroups and their basic characteristics are given in Tables 2 and 3.

#### 2.3.3. Functional Near-Infrared Spectroscopy

fNIRS is a practical technique that is frequently employed to estimate activation of the cortex through near-infrared probes [28, 29]. A continuous-wave NIRS instrument (Nirsmart, Danyang Huichuang Medical Equipment Co., Ltd., China) was utilized in this study. This system was equipped with 2 wavelengths of near-infrared light (730 nm and 850 nm) to detect changes in hemoglobin concentration in the cerebral cortex. This equipment has a total of 48 channels, including 23 emitters and 16 receivers. The instrument can measure total hemoglobin (HbT), HbO, and HbR concentrations.

A study [16] showed that there were extensive brain network connections between the prefrontal lobes and the thalamus and that the brain areas where conscious arousal was associated with. HbO was used as an evaluation indicator rather than HbR because the former is more sensitive in assessing cerebral blood flow [30, 31]. Therefore, in our study, HbO in the PFC was observed. We defined a PFC area containing 19 channels (channels 29/30/31/32/33/34/35/36/37/38/39/40/41/42/43/44/45/46/47).  Figure 2 shows the location of the channels corresponding to the PFC. In addition, the locations corresponding to channels 29, 30, 35, 36, 42, and 43 were artificially defined as right prefrontal cortex (R-PFC), the locations corresponding to channels 31, 32, 37, 38, 39, 44, and 45 as middle prefrontal cortex (M-PFC), and the locations corresponding to channels 33, 34, 39, 40, 41, 46, and 47 as left prefrontal cortex (L-PFC).

The article "Effects of Acupuncture on Cortical Activation in Patients with Disorders of Consciousness: A Functional Near-Infrared Spectroscopy Study" was published in 2022. Journal: Evid Based Complement Alternat Med.

### 2.4. Data Processing and Analysis

#### 2.4.1. fNIRS Data Processing

As the signal collected in fNIRS is susceptible to interference from external noise, we preprocessed the initial data with NirSprak. Data processing includes the following steps: selected the channels, we were interested in: prefrontal cortex; automatically eliminated the motional artefacts not relevant to this experiment; light intensity signal was converted into optical density (OD); the components with the frequency between 0.01 Hz and 0.2 Hz were filtered by using bandpass filtering [32, 33]; OD was transmitted into the concentration changes of HbO using modified Beer–Lambert law [34, 35]; and a hemodynamic response function (HRF) was obtained. The HbO values were applied to each of the analyses in this study.

#### 2.4.2. Analysis of Hemodynamic Response and Prefrontal Cortex Activation

The general linear model (GLM) is used in many fNIRS studies [36, 37]. After preprocessing, we applied GLM to implement an individual-level analysis channel by channel [38]. Afterward, a one-sample *t*-test was used on each channel to compare the HbO concentration between the resting state and acupuncture. A significance threshold (*P* < 0.05) was set and a false discovery rate (FDR) correction [39, 40] was performed. *P* value under 0.05 for a channel indicated a significant difference in HbO concentration between the resting state and during acupuncture, in which case the cortical area corresponding to that channel was considered to be activated. Then, the activation of the channels and their corresponding patterns of changes in the concentration of HbO in the cerebral cortex were observed.

#### 2.4.3. Cortical Functional Connectivity Analysis

In order to explore the mechanism of action of acupuncture to improve the impairment of consciousness, we used functional connectivity analysis to observe the effect of acupuncture on the functional connectivity of the cortical network. The changes in HbO concentrations at each time point measured by the subject during acupuncture manipulation and resting state were extracted in the network module of the NirSpark software, and the Pearson correlation coefficients [41] of the HbO and HbR contents of each channel were analyzed on a time series. The Fisher-*Z* transformation [42] was then performed, and the transformed values were defined as the functional connection strengths between the channels.

The article "Effects of Acupuncture on Cortical Activation in Patients with Disorders of Consciousness: A Functional Near-Infrared Spectroscopy Study" was published in 2022. Journal: Evid Based Complement Alternat Med.

#### 2.4.4. Analysis of the Correlation between Hemodynamic Response and Severity of DoC

After grouping according to GCS scores, it was found that the sample sizes of the moderate DoC and severe DoC groups differed significantly, and there was a significant difference (*P*=0.031) in age, so no further statistical analysis was done on this. Therefore, in this study, the hemodynamic responses of patients in the MCS and VS groups were analyzed and compared and then further investigated the potential relationship between the hemodynamic responses and the severity of DoC.

To explore the potential relationship between the severity of impaired consciousness and the hemodynamic response of the PFC, the data were processed as follows: select the data for the activated channels (channels 32, 34, 45, and 46) in the PFC; calculate the mean HbO concentration of the activated channels in the resting and acupuncture manipulation states and compare them to calculate the difference between the two; and two-sample *t*-test for changes in HbO concentration for each activated channel.

## 3. Results

In total, 16 patients (age: 60.75 ± 19.74 years; 7 males and 9 females) with DoC were enrolled in our study. The basic features of the subjects are given in Table 4.

### 3.1. Hemodynamic Response and Cortical Activation

The hemodynamic response of all patients was measured from the PFC area. In the present study, the change in HbO concentration was used as the main observational indicator representing cortical cerebral blood flow. Compared to baseline, all observed channels induced typical event-related changes in hemodynamic responses during needle twirl. It was found that the concentration of HbO in the PFC showed a tendency to increase during acupuncture manipulation, while the concentration of HbO decreased at resting state compared to baseline, suggesting that acupuncture of the Renzhong point could increase cerebral blood flow to PFC.  Figure 3 shows an example of the relative concentration changes of HbO of one subject during the block tasks.

Unfortunately, the study found that not all patients had the same activation channels, but several of all channels in the PFC were activated more frequently, which may be related to the patient's degree of arousal. In other words, it was found that changes in HbO concentration in some channels (channels 32, 34, 45, and 46) of the PFC were significantly increased during needle manipulation compared to baseline among more people (Figure 3). Besides, it was said that the four activated channels correspond to the L-PFC (channels 34 and 46) and M-PFC (channels 32 and 45). The specific location in the PFC corresponding to the activated channels is shown in Figure 4.

The article "Effects of Acupuncture on Cortical Activation in Patients with Disorders of Consciousness: A Functional Near-Infrared Spectroscopy Study" was published in 2022. Journal: Evid Based Complement Alternat Med.

### 3.2. Acupuncture Manipulation-Related Functional Connectivity

The functional connectivity diagram based on HbO concentration is shown in Figure 5. Almost all network connectivity diagrams showed a pattern that the connection strength of the L-PFC was generally higher than that of the right during acupuncture manipulation compared with the resting state. Importantly, the diagrams also clearly demonstrated that the L-PFC has distinctly increased functional connections with the M-PFC and left occipital lobe (LOL). Moreover, compared with the R-PFC, L-PFC and M-PFC were found to have slightly higher functional connectivity strength during acupuncture manipulation.

### 3.3. Correlation between the Changes in HbO Concentration and Severity of DoC

The HbO concentrations of different activated channels between the VS group and the MCS group were compared. The results showed that the mean HbO concentration of the 32 and 46 channels at the time of needle twirling in the VS group was higher than the MCS group, and there was no statistically significant difference (*P* = 0.740; *P* = 0.465). Meanwhile, the mean HbO concentration of the 34 and 45 channels in the VS group was lower than the MCS group, and there was also no significant difference (*P* = 0.532; *P* = 0.795). In addition, it was found that the changes in HbO concentration (the difference in HbO concentration between the acupuncture twirl state and the resting state) in the MCS and VS groups showed the same pattern as the mean HbO concentration. Overall, the differences in HbO concentration and mean HbO concentration of the four activated channels in the VS group were slightly higher compared to the MCS group, but the difference was not significant (Table5).

## 4. Discussion

Consciousness disorder is a common condition after brain injury. Although several studies [43–48] have suggested that acupuncture can effectively improve consciousness states, the therapeutic mechanism is not well understood. A previous study [49] showed that fNIRS could be applied to understand brain function in patients with DoC. However, no relevant literature involving patients with DoC was found on the effect of acupuncture on the hemodynamic response of the PFC with the monitor of the fNIRS system. The PFC may be a key site for regulating awareness and can be used to signal the emergence of consciousness [50, 51]. Furthermore, a study by Hong et al. [52] demonstrated that acupuncture could increase the activated area and enhance the connectivity in the PFC. Therefore, this study was the first to utilize fNIRS to measure the hemodynamic response of the PFC to investigate the effect of acupuncture on the hemodynamic response of the PFC in patients with impaired consciousness, to analyze the brain network functional connectivity, and to further explore the potential relationship between the hemodynamic response and the severity of DoC. For this purpose, 16 participants (6 MCS patients and 10 VS patients) received acupuncture treatment in a relatively quiet environment with fNIRS recording.

The article "Effects of Acupuncture on Cortical Activation in Patients with Disorders of Consciousness: A Functional Near-Infrared Spectroscopy Study" was published in 2022. Journal: Evid Based Complement Alternat Med.

Our results demonstrated that the prefrontal cortical concentration of HbO was visibly increased during the acupuncture manipulation phase and declined during the resting phase, compared with baseline. This phenomenon was somewhat consistent with the study by Zhang et al. [53], whose results suggested that HbT concentration in the PFC increased when patients received stimulation. Importantly, the effects of three acupuncture manipulation blocks on the concentration of HbO were fairly similar. Moreover, within each resting state, the concentration of HbO decreased from the end of the acupuncture manipulation to the next beginning of stimulation. These findings might imply that acupuncture may contribute to the restoration of the level of consciousness by participating in the neuromodulation of the prefrontal regions, especially the PFC locations corresponding to channels 32, 34, 45, and 46. It is highly likely that the excitability of the cortex corresponding to these four activated channels serves as a signal marker for the emergence of consciousness, and further studies need to be done in the future to confirm this idea. Furthermore, we observed more significant changes in the concentration of HbO in the L-PFC and M-PFC than in the R–PFC. That means cortical excitability in the left prefrontal and middle prefrontal may be important for the emergence of awareness.

In this study, we found that the connection strength of the L-PFC was generally higher than that of the right during acupuncture manipulation compared with the resting state. However, there were significant differences in the strength of functional connectivity between individuals. One possible reason for this is the wide variation in the age of the subjects included in this experiment, with the oldest being 91 years old and the youngest being 21 years old. The strength of functional connectivity may be largely related to the subject's age. A study by Chenyu et al. [54] proposed that the strength of functional brain connections is weaker in older adults compared to young adults. Interestingly, compared with the R-PFC, M-PFC and L-PFC were found to have slightly higher functional connectivity strength during acupuncture manipulation. This finding differs from the previous study by Leon-Dominguez et al. [55] who indicated that only the right dorsomedial PFC was significantly activated during the emergence phase. Further studies need to be done to distinguish the specific functions of the L-PFC as well as the right dorsomedial PFC.

The article "Effects of Acupuncture on Cortical Activation in Patients with Disorders of Consciousness: A Functional Near-Infrared Spectroscopy Study" was published in 2022. Journal: Evid Based Complement Alternat Med.

Our study found only a weak difference in hemodynamic responses of prefrontal areas between the VS and MCS groups. In other words, no significant correlation was found between the cortical hemodynamic response and the severity of DoC. Some previous articles have also attempted to investigate the hemodynamic differences between the MCS and VS groups, but no statistically significant differences were found. A review by Liberati et al. [56] also illustrated that half of the researchers reported statistically significant differences between VS and MCS patients. One reason for this may be that the data measured by fNIRS is influenced by the patient's systemic physiological state (such as heart rate, blood pressure, and respiratory rhythm) [57], resulting in a less than typical fNIRS response, increasing the incomparability of the patients' fNIRS response [58]. Another reason could be that the nociceptive stimuli produced during acupuncture manipulation influenced the fluctuations in patient wakefulness and masked the differences between the two groups.

There were three limitations in our study. The first limitation of this study was the technical challenge of using an fNIRS device. First, the number of optical channels used in this study is limited and does not completely cover all regions of the PFC; again, although the measured data have been subjected to a series of preprocessing, for example, automatic removal of motion artifacts and filtering algorithms, there are still effects that cannot be completely eliminated, which in turn affects the experimental results; finally, poor contact between the probe and the scalp may result in weak signal acquisition. Therefore, in future studies, a more advanced fNIRS instrument will need to be used to obtain more accurate results. Furthermore, greater processing methods will need to be utilized in further studies.

The second limitation of our study was the small sample size and the wide variation in the age of the subjects included in this experiment. It has been shown that the hemodynamic response of the cortex decreases with age, even in healthy adults [58]. Thus, in future studies, the hemodynamic response of patients with DoC at different ages can be analyzed separately, thus reducing the effects due to neurodegenerative changes.

The article "Effects of Acupuncture on Cortical Activation in Patients with Disorders of Consciousness: A Functional Near-Infrared Spectroscopy Study" was published in 2022. Journal: Evid Based Complement Alternat Med.

The third limitation of our experiment was that the hemodynamic response of patients in the resting state was not collected separately. The study was a block-designed experiment in which acupuncture stimulation was given for an extended time, followed by a period of resting state. With this approach, there may be a temporal lag effect of acupuncture on the hemodynamic response of the patient's cortex, resulting in the hemodynamic response during resting state not returning to the starting level and thus masking part of the effect of acupuncture on changes in the hemodynamic response. The hemodynamic response of patients in the resting state needs to be collected separately in subsequent studies.

Despite some limitations of our study, it is still instructive for clinical practice. This study may provide a reference for the mechanisms of improving awareness disorders by acupuncture, but its specific effects require further investigation. Furthermore, the potential of using the fNIRS device to detect the impact of acupuncture in patients with consciousness disorders is significant.

## 5. Conclusion

Our results showed that the concentration of HbO in PFC (especially in the L-PFC and M-PFC) was increased during the acupuncture manipulation phase and declined during the resting phase. In addition, we also observed the connection strength of the left cerebral cortex was generally higher than that of the right during acupuncture manipulation compared with the resting state. Finally, only a weak difference in hemodynamic responses of prefrontal areas between the VS and MCS groups was found, but no statistically significant differences. These results indicate that acupuncture can increase the concentration of HbO in the PFC (especially in the L-PFC and M-PFC) and strengthen the connection strength of the left cerebral cortex. Our findings suggest that there is no significant correlation between the cortical hemodynamic response and the severity of DoC.

## Figures and Tables

**Figure 1:** Block sequence of three tasks.

**Figure 2:** The cortical locations correspond to the channels. The area circled in red is the location of the prefrontal cortex (PFC).

**Figure 3:** The time-series response for concentrations of HbO in the four channels (channels 32, 34, 45, and 46) in the prefrontal cortex. The period in the red areas represents the acupuncture manipulation, while the white areas represent the resting state. This figure was generated with NirSprak software (developed by Danyang Huichuang Medical Equipment Co., Ltd., China).

The article "Effects of Acupuncture on Cortical Activation in Patients with Disorders of Consciousness: A Functional Near-Infrared Spectroscopy Study" was published in 2022. Journal: Evid Based Complement Alternat Med.

**Figure 4:** The activation maps with cortically projected channel positions.

**Figure 5:** Analysis of functional connectivity in two subjects with consciousness disorders during acupuncture manipulation. R-PFC, right prefrontal cortex; L-PFC, left prefrontal cortex; M-PFC, middle prefrontal cortex; PL, parietal lobe; R-TA, right temporoparietal association; L-TA, left temporoparietal association; ROL, right occipital lobe; LOL, left occipital lobe.

**Table 1:** CRS-R criteria for VS and MCS.

CRS-R subscales	VS	MCS
Auditory	≤2	3–4
	And	Or

Visual	≤1	2–5
	And	Or

Motor	≤2	3–6
	And	Or

Verbal	≤2	3
	And	Or

Communication	0	1–3

CRS-R, coma recovery scale-revised; VS, vegetative state; MCS, minimally conscious state.

**Table 2:** Characteristics of VS and MCS groups.

Features	VS group (*n* = 10)	MCS group (*n* = 6)	*P* value
Age (years)	56.2 ± 19.89	68.33 ± 18.62	0.356
Gender (M/F)	5M/5F	2M/4F	0.633
CRS-R (score)	3.1 ± 1.29	7.3 ± 1.37	0.001

CRS-R, coma recovery scale revise; VS, vegetative state; MCS, minimally conscious state; M, male; F, female.

**Table 3:** Characteristics of moderate and severe groups.

Features	Severe DoC group (*n* = 13)	Moderate DoC group (*n* = 3)	*P* value
Age (years)	55.62 ± 18.06	83.00 ± 7.21	0.031
Gender (M/F)	7M/6F	3F	0.213
GCS (score)	5.67 ± 1.50	9.25 ± 0.96	0.07

GCS, Glasgow coma scale; DoC, disorders of consciousness; M, male; F, female.

**Table 4:** The basic features of patients.

Patients	Age (years)	Gender	Disease duration (months)	Lesions	Medical history
01	47	Female	7.5	Pons, thalamus	Hypertension
02	44	Male	24	Brainstem	Hypertension
03	72	Male	4	Frontoparietal-temporal	No
04	72	Male	36	Right basal ganglion	Hypertension
05	55	Female	3	Brainstem	Hypertension
06	82	Female	2	Ruptured hemorrhage in the cavernous sinus segment of the right internal carotid artery	Hypertension
07	46	Male	2.5	Brainstem	Hypertension
08	42	Female	2.5	Brainstem, cerebellar	Hypertension
09	67	Male	1.5	Left basal ganglion, thalamus	Hypertension
10	81	Female	36.5	Right basal ganglion	Hypertension
11	53	Female	1	Right basal ganglion	No
12	91	Female	48	Multiple subcortical infarcts	Hypertension, diabetes
13	81	Female	16	Multiple subcortical infarcts	Hypertension, diabetes
14	21	Male	1.5	Ischemic-hypoxic encephalopathy	No
15	41	Male	1	Brainstem	Hypertension
16	77	Female	7.5	Frontoparietal-temporal	Hypertension, diabetes

**Table 5:** Comparison of HbO concentrations in different channels of the two groups (VS and MCS groups).

Channel	Mean HbO concentration at stimulation (mmol/L)			Difference HbO concentration (mmol/L)		
	VS group	MCS group	*P* value	VS group	MCS group	*P*value
32	0.061	0.043	0.740	0.086	0.044	0.430
34	0.062	0.083	0.532	0.071	0.096	0.501
45	0.062	0.072	0.795	0.077	0.078	0.972
46	0.049	0.026	0.465	0.057	0.048	0.775
Total	0.059	0.056	0.875	0.073	0.067	0.759

HbO, oxyhemoglobin; VS, vegetative state; MCS, minimally conscious state.

The article "Effects of Acupuncture on Cortical Activation in Patients with Disorders of Consciousness: A Functional Near-Infrared Spectroscopy Study" was published in 2022. Journal: Evid Based Complement Alternat Med.

## Additional Points

The concentration of HbO in PFC was increased during the acupuncture manipulation and declined during the resting state.
